The article "Construction and Computation of the College English Teaching Path in the Artificial Intelligence Teaching Environment" was retracted in 2023. Reasons: unreliable results or conclusions; concerns about the data; concerns about the peer review; concerns about the citations.

# Construction and Computation of the College English Teaching Path in the Artificial Intelligence Teaching Environment

**DOI:** 10.1155/2022/3415999

**Published:** 2022-09-30

**Authors:** Shaojie Liu

**Affiliations:** College of Foreign Languages, Shaanxi Xueqian Normal University, Xian, Shaanxi 710100, China

## Abstract

Today, English is the world's main international language and is widely spoken. In this context, the learning of English has long been valued by all countries. In addition, English plays an essential role in the process of economic globalization, specifically in the majority of countries where English is not the native language. At the same time, as China's integration into the world grows, the importance of English has become more pronounced, and the demand for English language skills has increased. At present, China's ever-expanding opening to the outside world, its developing science and technology, and its rising international status have created an urgent need for English-speaking professionals. This will lay the foundation for China's economic and social development and enable China to play a greater and more active role in international affairs, which has great practical and far-reaching historical significance. At present, the traditional English teaching mode has been criticized due to a great number of issues. At the same time, the new English language standards and the change of evaluation methods have created new demands on English teaching methods. As a result, with the development of artificial intelligence technology, the application of artificial intelligence technology in the field of education has brought new directions for the optimization of English classroom. In addition, diversified network technologies also provide new support for the realization of intelligent and collaborative English classroom teaching. To be specific, the maturity of English intelligent speech synthesis and intelligent speech evaluation technologies has enabled intelligent technologies to reach or even surpass the level of human teachers in certain areas. However, due to the limitations of the market environment and evaluation methods, the products that can focus on English classroom teaching are not highly intelligent and less collaborative. What is more, the process of English classroom intelligence has stagnated compared to other subjects. Obviously, from the perspective of integrating artificial intelligence technology with English classroom, it is quite necessary and feasible to design and develop an intelligent teaching assistant that can be applied to college English teaching. As information technology continues to evolve, both national and teacher levels are beginning to focus on how it can be better used in the teaching of subjects. Therefore, the use of online information technology in teaching and learning presents a great opportunity for research and practice in English language learning at the university level.

The article "Construction and Computation of the College English Teaching Path in the Artificial Intelligence Teaching Environment" was retracted in 2023. Reasons: unreliable results or conclusions; concerns about the data; concerns about the peer review; concerns about the citations.

## 1. Introduction

English is one of the major international languages spoken in the world today. What is more, English is the most widely spoken language in the world [1]. In other words, English occupies an important place in the process of economic globalization. In fact, the majority of countries place a high priority on the teaching of English [2, 3]. As China's integration into the world grows, its importance becomes more pronounced and the demand for English language skills becomes higher and higher. At the same time, China's expanding openness to the outside world, its advancing science and technology, and its growing international status have created an urgent need for English-speaking professionals [4]. This will lay the foundation for China's economic and social development and enable China to play a greater and more active role in international affairs [5]. As a result, the teaching of English becomes an important part of the basic education in China, and it is also one of the measures of the quality of a country's nationals. For today's college students, growing up in an open and tolerant era, learning English well means understanding the rich culture behind the language [6]. In addition, learning English gives college students a new way of seeing the world. At the same time, language is a bridge between us and another country. For example, while we are admiring the exoticism of another country, we can also use English to introduce the world to the glorious history and culture of China. This allows the world to gain a better understanding of China, and it enhances friendship between China and the rest of the world [7]. More importantly, learning English will help college students learn advanced science and technology from abroad, which will help China move forward more quickly. In order to achieve this goal, it is quite necessary to cultivate the comprehensive English application ability of college students [8]. First of all, it is necessary to improve students' English listening and speaking skills. After all, great English listening and speaking skills are positive for improving the overall quality of students in all aspects and laying a solid foundation for their future work as well as social interaction.

College English is a very crucial public course in higher education. To be specific, this kind of curriculum adopts English as the medium as well as language of instruction in order to promote general education [9]. As the most essential content of undergraduate foreign language education, college English has different characteristics from other courses [10]. It is only when its objectives, content, teaching activities, and assessment system fully reflect its unique requirements that it can truly achieve the ultimate goal of teaching this subject [11]. With the advent of the information age, global economic integration and international exchange are deepening in various industries and fields [12, 13]. The requirements for foreign language skills of professionals, especially English as an international language, are becoming more and more common, and the requirements for deeper English skills are becoming more prominent [14]. In international communication, the English intercultural communication ability of key personnel directly will also affect the process of international communication, science and technology exchange, and the smooth transition of cultural conflicts in various fields and even determines the ultimate success of project cooperation [15, 16]. The effective use of English and cross-cultural communication skills are very important.

The article "Construction and Computation of the College English Teaching Path in the Artificial Intelligence Teaching Environment" was retracted in 2023. Reasons: unreliable results or conclusions; concerns about the data; concerns about the peer review; concerns about the citations.

With the rapid development of information technology, people's learning environment and learning methods are constantly being enriched and improved [17]. In this context, various educational concepts and perspectives based on the information technology environment are also emerging and new. As a result, the combination of traditional teaching design and information technology is inevitable [18]. Therefore, in recent years, the reform of English teaching in universities has been transforming into network technology-based teaching. As shown in Figure 1, multimedia, tablets, cell phones, computers, as well as other information tools are flooding into college English classrooms as effective tools to support teachers' teaching and enrich college English teaching mode [19, 20]. In this context, with the support and assistance of such information technology environment, the shortcomings of the traditional college English teaching mode have been improved to a certain extent [21]. In other words, the original single plane teaching method has become more vivid and three-dimensional.

As shown in Figure 2, there are three main modes of teaching English in the university based on information technology environment. The first one is the group learning mode. This mode refers to the teacher's one-to-many teaching of students with the aid of IT equipment. This is also the most common mode of teaching English in college. To be specific, the teacher needs to teach the whole class through PPT and projection equipment [22]. The second mode is the individual learning mode, in which students choose and learn the course content independently through learning systems. The third is the blended learning model. This mode means that teachers use mobile devices as a medium to combine various learning modes such as group learning, independent learning, and social interactive learning in a hierarchical and organized manner through information technology to provide students with more diverse and rich learning options and learning styles [23]. The first and second modes of learning are the most commonly used in today's university English teaching. Their advantages are obvious, but their disadvantages cannot be ignored. In this context, a blended learning model that integrates mobile devices is particularly important [24]. Therefore, it is an important proposition to study the reform of college English teaching mode and promote the effective development of college English teaching by combining various teaching aspects such as group learning, independent learning, social sharing, and multiple evaluation in a hierarchical and organized way, and giving students a more free and efficient learning environment.

The article "Construction and Computation of the College English Teaching Path in the Artificial Intelligence Teaching Environment" was retracted in 2023. Reasons: unreliable results or conclusions; concerns about the data; concerns about the peer review; concerns about the citations.

Fragmented mobile learning has been a hot topic in recent years in teaching and learning research. The original idea of this concept is to enable learners to selectively separate learning content effectively through the use of mobile tools that transcend the constraints of time and space [25]. This allows learners to freely choose and control the content and timing of their learning and to extract meaningful pieces of knowledge from the vast amount of information available. Fragmented learning is an adaptation of learning styles to the fast-paced nature of modern life. It gives great freedom and independence to learning and deeply meets the modern people's need for free, efficient, and fast learning [26]. For this reason, in recent years, mobile tools such as microblogs, WeChat, and mobile APPs have been adapted to each other and jointly promoted fragmented learning. This can make fragmented mobile learning, i. e., learning in pieces through mobile tools, more popular [27]. The design of a blended university English teaching model cannot be achieved without the support of mobile tools. It allows learning to occur in fragments that are not limited to the classroom, thus giving students more freedom and choice. As a result, diversified network teaching environment has become a hot topic of research in college English classroom teaching.

Big data is ushering in a major transformation. Faced with the huge amount of information resources, people need to develop online learning behavior and habits with a new way of thinking [28]. The widespread use of mobile tools is profoundly changing the way people live and learn. The mobile learning and fragmented learning brought about by mobile tools make learning happen beyond the limitations of time and space, and moreover, it adapts to the learners' needs for learning autonomy and independence [29]. The immediacy and portability of mobile tools also provide new forms and carriers for the presentation and development of university English teaching resources. In other words, more teaching activities can be carried out and run with mobile tools as the scaffolding [30]. Therefore, combining mobile learning with university English courses is a choice that is in line with the trend of technological development and the development of the times. The application of mobile tools should be the key to the effective implementation of blended teaching and learning design and should be the focus of research on English classroom teaching.

The article "Construction and Computation of the College English Teaching Path in the Artificial Intelligence Teaching Environment" was retracted in 2023. Reasons: unreliable results or conclusions; concerns about the data; concerns about the peer review; concerns about the citations.

What is more, the use of a series of intelligent technology products in the English classroom has enriched the content as well as the mode of English classroom teaching [31]. To a certain extent, this mode has also improved the efficiency of English classroom teaching. However, the use of technology also limits teachers' own development. As a result, how to balance the roles of intelligent technology and teachers in the classroom and how to realize the human-computer collaborative teaching mode are important issues faced by the technology-enhanced classroom teaching. In order to address these issues, this study designs and develops an intelligent English teaching assistant from the perspective of human-computer collaborative teaching to solve the problems of speech input and language environment creation in English teaching [32]. The assistant has the main functions of text-to-speech, automatic speech evaluation, and listening materials creation. In addition, this study uses the intelligent teaching assistant to assist English teachers to carry out classroom teaching so as to solve a great number of problems in English teaching such as nonstandard speech input, promote the modernization and intelligence of English teaching, and realize the integration of artificial intelligence technology and English subject teaching.

## 2. Analysis of Learning Situation of College English Teaching

The design and implementation of the teaching process contains a great number of basic aspects and the synergy and influence of many factors need to be considered. As shown in Figure 3, in the process of teaching design and implementation, learners, teachers, teaching objectives, teaching contents, teaching media as well as some other factors are integrated in the whole teaching process. To be specific, they together form the basic structure of the teaching model. At the same time, the synergy of these factors ensures the proper implementation of teaching and learning. As a result, the discussion and analysis of these basic factors can facilitate the design and implementation of teaching and learning. In other words, it is only through a comprehensive and specific understanding of these basic factors that we can make proper judgment and design. In addition, the whole process of teaching and learning can be adjusted and modified according to what may happen.

The article "Construction and Computation of the College English Teaching Path in the Artificial Intelligence Teaching Environment" was retracted in 2023. Reasons: unreliable results or conclusions; concerns about the data; concerns about the peer review; concerns about the citations.

### 2.1. Learner Analysis

The learner is the main subject of instructional design and the center of the entire teaching and learning process. In addition, the learner is the starting and ending point for all instructional activities and arrangements. The characteristics of learners influence and guide the development of instructional a result, the analysis of learners should be placed before teaching. In fact, the majority of the learners for college English teaching are young students. These students are influenced by social, media, and family factors, and they have outstanding characteristics in behavior, emotion, thinking, and psychological cognition. At the same time, the rapid development of social economy and science and technology has provided them with a huge amount of information and the means to obtain it. This information can cultivate their active thinking, open personality, and broad vision. As a result, they form their own opinions and values on many issues early and even form their own cultural habits.

Cognitive development is the process by which an individual's ways of acquiring knowledge and skills and their ability to solve related problems change in stages over time. The most important factors that are emphasized are time and mechanism. It can be said that cognitive development represents, in part, the way learners understand the outside world, their thinking patterns, and their ability to learn. These competencies make it possible to design more contextualized instructional activities. After all, learners have a clear understanding of their place in the learning situation and their responsibilities. In addition, they are able to adapt more independently to changing learning processes free from the constraints of concrete experience. At the same time, they are able to find ways to adjust their own direction of inquiry as they work through problems. As a result, more cooperative and research-based learning can be applied in this process.

The article "Construction and Computation of the College English Teaching Path in the Artificial Intelligence Teaching Environment" was retracted in 2023. Reasons: unreliable results or conclusions; concerns about the data; concerns about the peer review; concerns about the citations.

### 2.2. Teaching Objective Analysis

Teaching objectives are specific, explicit statements of the visible behaviors that learners are expected to exhibit as a result of instruction. The original purpose of instruction is to enable learners to change in the direction specified by the goal. The teaching objectives set the direction of the instructional activity and guide the entire instructional process. During the teaching process, the teacher can control and regulate each step in the process. At the same time, the accomplishment of the teaching objectives is a test of the design and practice of the teaching activities. To be specific, the teacher can identify the issues and make corrections by comparing the final teaching results with the objectives set.  Figure 4 illustrates the categories of English training objectives in universities.

The content of a university English course is aggregated in the form of units, each of which is a specific topic. The various forms of content are organized under these themes and presented in detail under specific themes. Themes allow for the internal organization and connection of multiple forms and aspects of content. At the same time, these resources facilitate the learning of learners in various ways, such as visual, auditory, verbal, and practice, thus enriching the levels and forms of learning.  Figure 5 shows the content structure of university English course units. Course materials are the basic resources for teaching English at the university level, and units are the basic organizational units of university English course materials. The learning content is organized and aggregated in the form of thematic units. As chapter-based and coherent teaching materials, the units of a university English course textbook have a similar organizational structure. However, the textbook is adapted and modified in specific chapters so that the teaching becomes unified as well as clear.

### 2.3. English Specific Skill

The starting point and ultimate goal of learning a language and culture is to be able to recognize and use it well in daily study and work, and this is also true for learning the English language. The accumulation of a large number of words, the practice of listening and speaking, and the memorization of relevant grammatical knowledge are all aimed at the smooth and efficient use of English for one's own benefit. As a result, it is essential to acquire certain English skills for daily life, study, and work, as well as for answering exams. To be specific, it enables people to achieve their goals in a faster and more efficient way. In addition, it can lead to a more skillful learning process in which people develop their own learning habits and find the most appropriate learning path for themselves.  Figure 6 illustrates the specific structure of college English skills.

The article "Construction and Computation of the College English Teaching Path in the Artificial Intelligence Teaching Environment" was retracted in 2023. Reasons: unreliable results or conclusions; concerns about the data; concerns about the peer review; concerns about the citations.

The composition of English language is organized and presented in the form of words, sentences, paragraphs, and chapters, and in this way, it is increased and expanded in number and length. English language learning skills are empirical rules that learners discover over time. Specifically, it is a broad and individualized set of skills that exist in all aspects of English language learning. The learning of English language, like the learning of other languages and cultures, can be developed and refined in multiple dimensions: listening, speaking, reading, writing, and translating. Therefore, the role of English language learning skills is to facilitate learners' effective and practical mastery and understanding of the formal content of words, sentences, paragraphs, texts, and chapters in the dimensions of listening, speaking, reading, writing, and translating.

## 3. Application of Diversified Network Teaching

The teaching design behavior mainly includes the design of teaching objectives, teaching methods, the development of curriculum resources, and collective lesson planning. Quality teaching resources are the basic guarantee of teaching effectiveness, and the design of English classroom requires the support of various media materials such as sound, text, and images. At present, English teachers mostly use PPT classroom materials to design teaching activities. Therefore, the production of PPT materials has become an inevitable part of every English teacher's lesson preparation, which undoubtedly brings great teaching pressure to English teachers. In traditional teaching, there are two ways for teachers to obtain audio materials. The first is the audio materials accompanying the textbook, and the second is the audio materials recorded by teachers themselves. The use of audio materials can ensure the quality of audio, but it lacks flexibility.

### 3.1. Network Structure Model Design

The C/S model assigns the system tasks to the client and server according to the rules and uses the cooperation between the client and server to accomplish the system tasks. The C/S model has the advantages of fast response time and strong security, but the development and maintenance costs are high, and it does not have cross-platform capability. To be specific, it mainly applies the browser to act as the client and puts the main task processing into the server. The B/S model has the advantages of cross-platform, no client maintenance, and easy development. However, this model also has the disadvantages of slow response time and lack of personalization. From the practical point of view of practicality, intelligence, and convenience, the English subject intelligent teaching assistant is implemented in the B/S mode. The user can access the server through a common browser, and the client can realize the relevant functions. This model reduces the requirements for the client, and the core functions depend mainly on the server to run, thus reducing the need for hardware conditions. As a result, access to the assistant can be achieved by installing a browser on the running computer. This simplifies the development, use, and maintenance of the assistant and also greatly improves system compatibility. The overall structure design and architecture logic of the intelligent teaching assistant is shown in Figure 7.

The article "Construction and Computation of the College English Teaching Path in the Artificial Intelligence Teaching Environment" was retracted in 2023. Reasons: unreliable results or conclusions; concerns about the data; concerns about the peer review; concerns about the citations.

The intelligent teaching assistant adopts B/S architecture. Therefore, teachers and administrators can access the system functions of Intelligent Teaching Assistant conveniently and quickly at any time and any place through the campus network. While completing intelligent teaching and management, it can also effectively ensure user information security. Users access the server through the browser, and the data exchange is done directly with the server. After that, the data in the database can be accessed through the server. This can effectively avoid the user's direct manipulation of the data in the database, thus making the user request relatively independent from the database. As a result, data security, reliability, and accuracy are guaranteed.

### 3.2. Module Design and Analysis

According to the concept of multimedia teaching, not only text but also graphics, illustrations, icons, video animation, audio, and other information media are needed in English teaching. In addition, it is necessary to use scientific technology to combine these media in a unified way. The design and creation of courseware provides teachers with the ability to quickly design activities and present content visually. To be specific, this function can effectively combine multiple teaching media to achieve a uniform and fast presentation of teaching content. The intelligent courseware editing and creation function should reflect the teacher's dominant position. As an intelligent tool for collaborating with teachers to design teaching activities, the assistant can be used to create intelligent courseware easily and quickly by intelligent means. On the basis of this, it can have the intelligent voice integration function, which is not available in traditional slides so that teachers can free themselves from the heavy workload of creating courseware and focus on classroom organization and management, activity design, as well as teaching reflection.

The article "Construction and Computation of the College English Teaching Path in the Artificial Intelligence Teaching Environment" was retracted in 2023. Reasons: unreliable results or conclusions; concerns about the data; concerns about the peer review; concerns about the citations.

The smart courseware editing feature is used by teachers to create multimedia web pages for classroom use. With the built-in visual web authoring tool, teachers can store the created pages in the cloud database. At the same time, they can use the browser to render the visual content of the web page when they use it. In this way, intelligent web pages can be created that provide a multidimensional display of English text in a randomized point-and-click manner. The intelligent voice courseware contains all the content that can be included in a web page. As a result, text, images, audio, video, tables, and other teaching materials can be inserted. In addition, it also has the functions of setting font and font size, setting image size, setting background color, and hyperlinks, etc.[33]

## 4. Conclusion

Unlike the traditional university English resource model, the university English teaching resource model in the context of multiple networks considers the relevant functions and characteristics of mobile tools. Specifically, it enables students to participate in the accumulation and improvement of teaching resources without the use of functions. As a result, teachers are no longer the only source of resource materials, and students are able to participate and interact more through the provision and sharing of resources. The flow of teaching resources is no longer a one-way process from teachers to students, but a mobile tool that allows more people to participate in the process of resource generation. The resource material is expanded and fed back in the cycle, and the release of relevant content can be the source of new feedback. As a result, resources are added in this circular pattern. At the same time, the resource structure is no longer only a medium for providing relevant materials but also a platform for mutual communication.

However, because there are few public resources, teachers still need to design and create their own intelligent voice courseware although the Intelligent Teaching Assistant provides a public resource library. As a result, there are fewer resources that can be directly used by teachers. As AI technology advances and intelligent teaching continues to evolve, the impact on the English classroom will deepen. The researchers and developers are still facing serious challenges, and the optimization and improvement of the shortcomings in this study will be part of the author's future research work.

## Figures and Tables

**Figure 1:** Teaching tools of college English teaching.

**Figure 2:** Mode of college English teaching.

**Figure 3:** Factors in the process of teaching design and implementation.

The article "Construction and Computation of the College English Teaching Path in the Artificial Intelligence Teaching Environment" was retracted in 2023. Reasons: unreliable results or conclusions; concerns about the data; concerns about the peer review; concerns about the citations.

**Figure 4:** Categories of English training objectives in universities.

**Figure 5:** Content structure of university English course units.

**Figure 6:** Specific structure of college English skills.

**Figure 7:** Structure design and architecture logic of the intelligent teaching assistant.

## Data Availability

The labeled dataset used to support the findings of this study are available from the corresponding author upon request.
